The article "FGF5 is expressed in melanoma and enhances malignancy in vitro and in vivo" was published in 2017. Journal: Oncotarget.

# FGF5 is expressed in melanoma and enhances malignancy *in vitro* and *in vivo*

**DOI:** 10.18632/oncotarget.21184

**Published:** 2017-09-23

**Authors:** Sara Ghassemi, Katharina Vejdovszky, Emine Sahin, Lukas Ratzinger, Karin Schelch, Thomas Mohr, Barbara Peter-Vörösmarty, Jelena Brankovic, Andreas Lackner, Alexandra Leopoldi, Diana Meindl, Christine Pirker, Balazs Hegedus, Brigitte Marian, Klaus Holzmann, Bettina Grasl-Kraupp, Petra Heffeter, Walter Berger, Michael Grusch

**Affiliations:** ^1^ Institute of Cancer Research, Department of Medicine I, Comprehensive Cancer Center Vienna, Medical University of Vienna, Vienna, Austria; ^2^ Translational Thoracic Oncology Laboratory, Division of Thoracic Surgery, Department of Surgery, Comprehensive Cancer Center Vienna, Medical University of Vienna, Vienna, Austria; ^3^ Department of Thoracic Surgery, Ruhrlandklinik, University Clinic Essen, Unversity of Duisburg-Essen, Duisburg, Germany

**Keywords:** FGF5, fibroblast growth factor, melanoma, malignant growth

## Abstract

Although FGF5 mRNA was previously found expressed in some melanoma cell lines in contrast to normal human melanocytes, neither its contribution to melanoma growth nor its expression in melanoma tissue has been investigated. Here we demonstrate that ectopic overexpression of FGF5 in human melanoma cells with low endogenous FGF5 expression increased clonogenicity and invasion but not short-term growth *in vitro*. Silencing of FGF5 in melanoma cells with high endogenous FGF5 expression had the opposite effect on clonogenicity. FGF overexpression led to increased signaling along the MAPK and NFAT axis but had no effect on STAT3 signaling. In an *in vivo* experiment in immunocompromised mice, human melanoma xenografts overexpressing FGF5 showed enhanced tumor growth, a higher Ki-67 proliferation index, decreased apoptosis and enhanced angiogenesis. Immunohistochemistry performed on a tissue microarray demonstrated FGF5 protein expression in more than 50% of samples of melanoma and benign nevi. These data suggest that FGF5 has oncogenic potential in melanoma cells and contributes to melanoma growth in a subset of patients. This highlights the importance of further evaluating FGF5 as potential biomarker and therapy target in melanoma.

## INTRODUCTION

Melanoma originates from pigment-producing melanocytes and its incidence has risen significantly in past decades. Although the development of immunotherapeutics like ipilimumab or pembrolizumab and of drugs targeting mutated BRAF like vemurafenib or dabrafenib has improved treatment options and survival for melanoma patients [1, 2], the curative treatment of advanced melanoma still remains a challenging future goal [3]. Identification of additional factors that contribute to melanoma progression and may provide novel targets for therapeutic agents is therefore still an important requirement to improve the outlook for melanoma patients.

The article "FGF5 is expressed in melanoma and enhances malignancy in vitro and in vivo" was published in 2017. Journal: Oncotarget.

Fibroblast growth factors (FGF) constitute a family of 18 polypeptides that transduce signals through receptor tyrosine kinases (RTK) named fibroblast growth factor receptors (FGFRs) 1 to 4. Signal transduction occurs along the mitogen-activated protein kinase (MAPK), the phosphatidylinositol-3 kinase (PI3K), the phospholipase Cγ (PLCγ), and the signal transducer and activator of transcription (STAT) pathways [4]. Several FGFs play crucial roles in embryonic development and are involved in wound healing and tissue maintenance [5]. However, overexpression, amplification or mutation of FGFs or FGFRs also contributes to malignancy in numerous tumor types. Amplification of FGFR1 occurs for instance, in non small cell lung cancer (NSCLC) [6] and breast cancer [7], while mutations of FGFR3 are found in bladder and cervix carcinoma [8]. Overexpression of FGFs was reported, for instance, for FGF8 and FGF19 in hepatocellular carcinoma (HCC) [9, 10] and for FGF2 in multiple cancers including melanoma and mesothelioma [11, 12].

FGF5 was first identified [13] by a screening approach for transforming oncogenes and later characterized as a major regulator of hair growth in mammals [14–16]. FGF5 deletion in mice leads to an angora phenotype [17] and FGF5 mutations are associated with trichomegaly in humans [18]. Investigations of oncogenic functions of FGF5 are relatively sparse so far. Increased expression of FGF5 was associated with pancreatic cancer [19], and high FGF5 expression was found in cell lines from renal cell carcinoma (6 of 10) prostate cancer (2 of 3) and breast cancer (1 of 2) [20]. Another study linked high TGFβ2 and FGF5 expression to NFkappaB activation in tumor cell lines from various malignancies including prostate and cervix cancer [21]. More recently, FGF5 was identified as a critical target of the tumor suppressive microRNA-188-5p in hepatocellular carcinoma [22]. In a previous study, we demonstrated oncogenic activity of FGF5 in astrocytic brain tumors, which could be attributed to both autocrine effects on the tumor cells as well as paracrine effects on endothelial cells [23]. With respect to melanoma, we and other groups have previously observed FGF5 expression in some melanoma cell lines in contrast to normal melanocytes, where FGF5 is hardly detectable [24, 25]. Despite these initial findings in melanoma cell lines and the proposed tumor-promoting role of FGF5 in other malignancies, FGF5 has not been further investigated in melanoma so far. Therefore, we asked whether FGF5 is expressed in human melanoma tissue and whether FGF5 expression may contribute to the malignant behavior of melanoma cells. In the current study, we demonstrate that FGF5 expression contributes to the malignancy of melanoma cells *in vitro* as well as in a mouse xenotransplant model and show that FGF5 protein is expressed in a considerable fraction of human melanoma tissue samples.

The article "FGF5 is expressed in melanoma and enhances malignancy in vitro and in vivo" was published in 2017. Journal: Oncotarget.

## RESULTS

### FGF5 is strongly overexpressed in more than one-third of melanoma cell lines

To select appropriate cell models, we initially screened normal human melanocytes and a panel of 28 human melanoma cell lines for FGF5 gene expression by qPCR. Cell line characteristics are shown in Table 1. In agreement with previous results [24, 25], FGF5 expression was hardly detectable in the normal melanocytes. In 12 of 28 melanoma cell lines in contrast, FGF5 was highly expressed (> 50-fold compared to normal melanocytes) (Figure 1).

**Table 1:** Histological classification, origin and mutation status of BRAF and NRAS of the cell lines used in the study [41]

Cell line	Classification^*^	Origin^**^	BRAF^V600E***^	NRAS^Q61***^
VM2	NM	PT	mut/wt	wt
VM10	SSM	PT	mut	wt
VM19	SSM	PT	mut/wt	wt
VM21	NM	PT	mut	wt
VM23	NM	PT	mut/wt	wt
VM25	NM	PT	mut/wt	wt
VM30	SSM	PT	mut	wt
VM32	NM	PT	mut/wt	wt
VM44	SSM	PT	mut/wt	wt
VM7	NM	PT	mut/wt	wt
VM1	SSM	LN	mut/wt	wt
VM5	SSM	LN	mut	nd
VM6	NM	LN	mut	nd
VM8	NM	LN	mut/wt	wt
VM15	uk	LN	wt	mut/wt
VM24	NM	LN	mut	wt
VM31	NM	ME	mut/wt	wt
VM9	SSM	Bone	wt	mut/wt
VM22	NM	Bone	mut/wt	wt
VM28	uk	Brain	mut/wt	wt
VM46	NM	Brain	mut/wt	wt
VM47	NM	Brain	wt	wt
VM48	NM	Brain	mut	wt
VM51	uk	Brain	mut/wt	wt

^*^ Histology of the primary tumor: NM, nodular melanoma; SSM, superficial spreading melanoma; uk, unknown primary lesion. ^**^Establishment of cell lines from primary tumors (PT), metastases (LN, lymph node; SC, bone; brain) and malignant effusions (ME) of malignant melanoma. ^***^wt, homozygous, only wild type allele detected; mut, homozygous, only mutant allele detected; mut/wt, heterozygous, both wild type and mutant allele detected; nd, not determined.

**Figure 1:** FGF5 is overexpressed in melanoma cell lines FGF5 expression in normal melanocytes (Norm Mel) and melanoma cell lines was determined by qPCR and normalized to the house-keeping gene beta 2 microglobulin. Expression in melanoma cell lines is depicted as fold expression compared to Norm Mel (set as 1). Twelve of 28 melanoma cell lines (43%) had more than 50-fold (red dotted line) elevated FGF5 gene expression levels compared to Norm Mel.

### FGF5 increases clonogenicity and invasion of melanoma cells *in vitro*

To analyze a potential contribution of FGF5 to malignant growth of melanoma cells, we ectopically expressed human FGF5 in two cell lines, VM1 and VM21, with low endogenous FGF5 levels. We used a bicistronic vector that enabled a dual selection for neomycin resistance and GFP expression. When analyzed by qPCR, FGF5 stable transfectants expressed about 800- (VM1-FGF5) and 600- (VM21-FGF5) fold increased FGF5 levels compared to the respective vector controls (VM1-GFP, VM21-GFP), thus achieving expression levels comparable to the high endogenous FGF5 expression levels observed in VM7 and VM8. When *in vitro* growth curves were established for VM1-FGF5 and VM21-FGF5 under standard growth conditions, no difference was observed compared to VM1-GFP and VM21-GFP, respectively (Figure 2A). However, when cells were seeded at low density to analyze clonogenicity, VM1-FGF5 cells but not VM21-FGF5 cells showed significantly increased colony formation (Figure 2B). In three additional cell lines (VM9, VM28 and A375) with low endogenous FGF5 expression, significantly increased clonogenicity was found upon treatment with FGF5 (Figure 2C). In an *in vitro* invasion assay, VM1-FGF5 cells also showed an increased ability to migrate through a collagen-coated porous membrane (Figure 2D) indicating that FGF5 leads to increased invasiveness in this cell model.

The article "FGF5 is expressed in melanoma and enhances malignancy in vitro and in vivo" was published in 2017. Journal: Oncotarget.

**Figure 2:** FGF5 enhances *in vitro* clonogenicity and invasion but not proliferation of melanoma cells with low endogenous FGF5 expression **(A)** VM1 (left panel) or VM21 (right panel) cells stably expressing FGF5 or the respective control cells (Contr) were grown in medium with 10% FBS and cell number was determined every 2^nd^ day. **(B)** VM1 (left panel) or VM21 (right panel) cells were seeded at low density in medium with 10% FBS and clonogenicity was determined after two weeks. **(C)** VM9, VM28 and A375 cells were seeded in medium with 10% FBS at low density and treated with FGF5 (10 ng/ml) or vehicle every third day. Clonogenicity was determined after two weeks. **(D)** VM1 cells stably expressing FGF5 or the respective control cells were seeded into collagen-coated transwell chambers and invasion through the collagen layer to the bottom of the well was determined after 72 h. ^*^ p < 0.05, ^**^ p < 0.01, ^***^ p < 0.001 FGF5 versus Contr, unpaired t-test.

### Knock-down of high FGF5 expression impairs clonogenic growth of melanoma cells

In the reverse approach, we tested whether knock-down of FGF5 in melanoma cells with high endogenous FGF5 expression would reduce their growth capacity. Four commercially available lentiviruses expressing shRNAs targeting FGF5 (shFGF5) were tested in VM8 cells for stable FGF5 knock-down compared to a non-silencing control lentivirus (shScr). The construct shFGF5-1 achieved the highest knock-down efficiency (Figure 3A) and was used for the subsequent experiment. In clonogenic assays, shFGF5-1 reduced colony formation of VM8 cells by 25% compared to shScr (Figure 3B). Comparable results were obtained when VM8 cells and VM47 cells, another cell line with high endogenous FGF5 expression, were transiently transfected with FGF5-targeting siRNA compared to non-silencing control siRNA that resulted in FGF5 knock-down efficiencies of 60% and 75% in VM8 and VM47, respectively (Figure 3C and 3D). As expected, the effect of silencing FGF5 could be reversed by addition of exogenous FGF5.

The article "FGF5 is expressed in melanoma and enhances malignancy in vitro and in vivo" was published in 2017. Journal: Oncotarget.

**Figure 3:** Silencing of FGF5 reduces *in vitro* clonogenicity of melanoma cells with high endogenous FGF5 expression **(A)** Lentiviral transduction with shFGF5-1 achieves strong silencing of FGF5 mRNA in VM8 melanoma cells. VM8 melanoma cells were stably transduced with lentiviruses expressing FGF5-targeting short hairpin RNAs (shFGF5-1 to shFGFR5-4) or scrambled control RNA (shScr). FGF5 transcript levels were determined by qPCR and are depicted as fold expression of the non-silencing control. VM8 cells stably expressing shFGF5-1 were used for the subsequent experiment. **(B)** VM8 cells with silenced FGF5 (shFGF5-1) and VM8 cells expressing non-silencing shRNA (shScr) were seeded at low density in medium with 10% FBS and clonogenicity was determined after 14 days. Bar graphs (left) and representative wells (right) are shown. **(C)** VM8 and VM47 cell were transfected with siRNA targeting FGF5 (siFGF5) or non-silencing siRNA (siNs) and FGF5 transcript levels were determined by qPCR. **(D)** VM8 cells and **(E)** VM47 cells were transfected with siNs and siFGF5 or transfected with siFGF5 in the presence of 10 ng/ml exogenous FGF5 (siFGF5+). ^*^ p < 0.05, ^***^ p < 0.001 sh/siFGF5 versus shScr/Ns, unpaired t-test (B), one-way ANOVA with Dunnets post-test (D, E).

### FGF5 expression affects MAPK and NFAT signaling

To explore potential signaling pathways that could be affected by FGF5 expression, we used reporter gene assays for the MAPK pathway, NFAT (nuclear factor of activated T-cells) and STAT3 signaling. VM1-FGF5 and VM21-FGF5 both showed significantly higher activity of MAPK and NFAT signaling than the respective GFP controls (Figure 4A). In contrast, STAT3 transcriptional activity showed rather a tendency to be decreased, which however was not statistically significant. A similar tendency towards decreased signaling was observed upon silencing of FGF5 in the VM8 cell line. NFAT signaling was below the assay detection limit in this cell model and STAT3 transcriptional activity was unchanged compared to the control (Figure 4B).

The article "FGF5 is expressed in melanoma and enhances malignancy in vitro and in vivo" was published in 2017. Journal: Oncotarget.

**Figure 4:** Reporter gene assays indicate increased transcriptional activity of the MAPK and NFAT but not the STAT3 axis in FGF5 overexpressing melanoma cells **(A)** VM1-FGF5 and VM21-FGF5 and the corresponding GFP controls were transfected with reporter constructs for MAPK, NFAT and STAT3 and transcriptional activity was determined after 24 h. **(B)** VM8 cells were co-transfected with siFGF5 or siNs (as control) and reporter constructs for MAPK and STAT3 and transcriptional activity was determined after 48 h. ^*^ p < 0.05, ^**^ p < 0.01 FGF5 versus Contr, one-way ANOVA with Bonferroni post-test.

### FGF5 overexpression increases tumor growth and proliferation rate *in vivo*

To test the impact of FGF5 overexpression on melanoma growth *in vivo* in a human to mouse xenotransplantation experiment, the cell line VM21 was used, due to its faster and more robust *in vivo* growth. VM21-FGF5 and VM21-GFP were subcutaneously implanted into severe combined immunodeficient (SCID) mice. VM21-FGF5 tumors were detectable earlier and grew more rapidly, reaching more than twice the volume of VM21-GFP tumors after 40 days (Figure 5A and 5B) at which time the mice were sacrificed and tumors excised and embedded for histological examination. Immunohistochemical (IHC) staining of formalin-fixed paraffin embedded (FFPE) tumor sections from the excised xenotransplanted tumors confirmed overexpression of FGF5 on the protein level in VM21-FGF5 compared to VM21-GFP cells and demonstrated the specificity of the antibody on paraffin sections (Figure 5B). Moreover, VM21-FGF5 tumors showed an enhanced rate of proliferating cells based on Ki67 index compared to VM21-GFP tumors (Figure 5C).

**Figure 5:** FGF5 enhances tumor growth and proliferation index *in vivo* **(A)** VM21 cells stably expressing FGF5 or control cells (Contr) expressing only GFP were injected subcutaneously into SCID mice (4 per group) and tumor volume (means ± SEM) was determined over 40 days before mice were sacrificed. **(B)** Representative examples of gross appearance of control and FGF5-overexpressing tumors (upper panels, scale bar = 1 mm) and of FGF5 protein expression determined by immunohistochemistry on formalin-fixed and paraffin-embedded tumor sections (lower panels, scale bar = 25 μm). **(C)** Percentage (upper panel) and representative examples (lower panels, scale bar = 25 μm) of Ki67-positive nuclei in FGF5-overexpressing and control tumors. **(D)** Percentage (upper panel) and representative examples (lower panels, scale bar = 100 μm) of apoptotic nuclei in histological sections of FGF5-overexpressing and control tumors. **(E)** Representative immunoblot of FGF5 in supernatants of control and FGF5 overexpressing VM21 cells. B2mg was used as control for sample loading **(F)** Quantitation (upper panel) and representative examples (lower panels, scale bar = 150 μm) of CD31-positive vessels in FGF5-overexpressing and control tumors. ^*^ p < 0.05, ^**^ p < 0.01, ^***^ p < 0.001 FGF5 versus Contr, unpaired t-test.

The article "FGF5 is expressed in melanoma and enhances malignancy in vitro and in vivo" was published in 2017. Journal: Oncotarget.

### FGF5 overexpression decreases apoptosis and increases angiogenesis *in vivo*

To further analyze potential mechanisms that could contribute to the increased growth of FGF5 overexpressing tumors, histological sections from the xenotransplantation experiment were used for apoptosis detection. VM21-FGF5 tumors showed decreased apoptosis rates when compared to VM21-GFP tumors (Figure 5D). Since VM21-FGF5 cells secrete an enhanced amount of FGF5 (Figure 5E), the tumor microenvironment could also contribute to the increased growth of VM21-FGF5 tumors. Indeed, CD31 staining of blood vessels, demonstrated a higher microvessel density in VM21-FGF5 tumors than in VM21-GFP tumors (Figure 5F).

### FGF5 is expressed in human melanoma tissue

To rule out the possibility that endogenous FGF5 expression occurs only in melanoma cell lines under culture conditions and may thus represent a cell culture artefact, we investigated FGF5 protein expression by IHC in a tissue microarray of human melanoma specimens. To ensure specificity of the staining, we used the same antibody that had shown enhanced staining intensity in the FFPE sections from FGF5-overexpressing xenografted tumors compared to the control tumors. Positive FGF5 immunoreactivity was detected in 14 of 23 benign nevi (61%) 36 of 56 primary melanomas (77%) and 13 of 20 metastatic melanomas (75%) (Figure 6A and 6B). The fact that FGF5 is present in about 60% of benign nevi and in an even higher percentage of primary melanoma, but is not further enhanced in metastatic compared to primary melanoma suggests that - similar to BRAF mutations [26] – FGF5 expression may be an early event in melanoma development and less important once metastasis has occurred. Data downloaded from the Cancer Genome Atlas (TCGA) further support FGF5 expression in tumor tissue from subsets of human melanoma patients (Figure 6C).

**Figure 6:** FGF5 is expressed in human melanoma tissue **(A)** FGF5 staining of a human melanoma tissue array was scored as absent, strong or weak in 23 benign nevi, 56 primary melanomas (Mel Prim) and 20 melanoma metastases (Mel Met). **(B)** Representative images of strong FGF5 staining (α-FGF5) and the respective non-immune serum control (Neg Contr) in a case of primary melanoma. Scale bar = 20 μm. **(C)** HTSeq Data were downloaded from the Cancer Genome Atlas (TCGA) using the TCGAbiolinks package and R [44]. Counts were normalized by library size.

The article "FGF5 is expressed in melanoma and enhances malignancy in vitro and in vivo" was published in 2017. Journal: Oncotarget.

## DISCUSSION

Our results are consistent with the notion that in addition to activation of the MAPK pathway by mutations of BRAF or NRAS in roughly 60% of melanoma patients [27], also over-activation of the FGF axis contributes to melanoma growth [28, 29]. In line with this, we have previously shown that combined inhibition of BRAF and FGFR1 has synergistic anti-melanoma effects [25]. Of note, FGF5 overexpression further enhanced MAPK pathway activity despite the presence of BRAF^V600E^ in both cell models. Enhanced NFAT activity in FGF5 overexpressing cells could be a consequence of FGFR1-mediated PLCγ activation as previously reported [30] and could contribute to enhanced melanoma growth via an anti-apoptotic activity [31]. In the past, most studies on FGFs in melanoma have concentrated on FGF2 [28, 32] and while - in addition to FGF2 - overexpression of FGF5 mRNA was noted in some melanoma cell lines more than two decades ago [24], FGF5 protein expression in melanoma tissue and its impact on melanoma growth were never investigated. Thus, we provide the first demonstration that FGF5 is expressed in melanoma tissue and, moreover, may support clonogenic survival and invasion *in vitro* and tumor growth in an *in vivo* model. FGFR1, the predominant receptor for FGF5, is abundantly expressed in melanoma cells [25] and likely is responsible for transducing autocrine stimulation by FGF5. Recently, we found highly elevated FGF5 expression also in 2 of 9 cell lines from malignant pleural mesothelioma [12], an asbestos exposure-related malignancy where FGFR1 expression is strongly associated with malignant growth and where FGF/FGFR-targeting treatment strategies are explored in clinical trials [12, 33, 34]. Thus, FGF5 overexpression may define specific subsets of tumors from different tissue origins. In cholangiocarcinoma cell lines, FGF5 was recently implicated in activation of the Hippo pathway and it was suggested that Hippo pathway activation, assessed *via* YAP expression, could serve as potential biomarker to identify patients with a higher likelihood of responding to therapies targeting the FGF/FGFR axis [35]. In colorectal carcinoma in contrast, FGF5 was one of 23 genes showing elevated DNA methylation in >50% of cancer tissue compared to non-neoplastic tissue [36]. While it was suggested that these genes could be used in diagnostic tests, the functional consequences of elevated FGF5 DNA methylation in colorectal cancer have not been explored at present.

In addition to autocrine effects on the tumor cells, FGF5 secretion by melanoma cells may have paracrine effects on endothelial cells and/or tumor-associated fibroblasts. This would be in agreement with our previous data in glioblastoma, where FGF5 enhanced proliferation and tube formation of endothelial cells [23] and related data in colorectal carcinoma, where tumor cell-secreted FGF18 increased the proliferation of endothelial cells and fibroblasts [37]. Recently, endogenously expressed FGF5 was shown to be an important promoter of angiogenesis in human aortic endothelial cells in an *in vitro* angiogenesis model [38]. The increased microvessel density in the FGF5 overexpressing tumors found in our study is in line with these data and could contribute to the faster growth and diminished apoptosis rate in these tumors due to improved oxygen and nutrient supply. The fact, that VM21-GFP had a clear growth advantage *in vivo* but not *in vitro* suggests a critical role of the tumor microenvironment in this model.

The article "FGF5 is expressed in melanoma and enhances malignancy in vitro and in vivo" was published in 2017. Journal: Oncotarget.

In summary, we show for the first time the expression of FGF5 protein in a substantial fraction of nevus and melanoma tissues and provide evidence for pro-tumorigenic functions of FGF5 in melanoma. Our findings warrant future studies investigating whether FGF5 expression correlates with tumor grade, clinical disease outcome or therapy response in melanoma and whether FGF5 overexpression in melanoma cells may be indicative of a precursor/stem cell phenotype as suggested by its presence in neuronal precursor cells [39].

## MATERIALS AND METHODS

### Cell culture

Melanoma cell lines were established from surgical specimens of primary or metastatic melanoma as previously described [40]. Cells were grown in RPMI 1640 medium with 10% FBS under standard conditions (37°C, 5% CO_2_). Classification, origin and mutational status of BRAF and NRAS are shown in Table 1. Data were obtained as previously published [41]. In addition, the melanoma cell lines A375, A2058, SK-MEL-28 (all harboring the BRAF^V600E^ mutation and wild type NRAS) and MEWO (wild type for BRAF and NRAS) were obtained from ATCC (Manassas, VA, USA) and cultured in DMEM with 10% FBS. Cell lines were authenticated by array comparative genomic hybridization (aCGH) and regularly checked for *Mycoplasma* contamination. Normal human melanocytes (Norm Mel) were from Lonza (Basel, Switzerland) and were cultured according to the supplier´s instructions.

### Quantitative real-time PCR (qPCR)

Total RNA from logarithmically growing cells was isolated with TRIzol reagent (Thermo Scientific, Waltham, MA, USA) and 2 μg RNA per sample were reverse transcribed with MMLV reverse transcriptase (Thermo Scientific). One μl cDNA, corresponding to 50 ng RNA, was analyzed per PCR. Quantitative real-time PCR (qPCR) was performed with Taqman assays for FGF5 (Hs00170454_m1, Applied Biosystems, Foster City, CA, USA) and beta 2 microglobulin (b2mg, Hs99999907_m1, used as reference) on an ABI Prism 7500 thermocycler. Semiquantitative determination of gene expression was performed by applying the 2^(−ΔΔCT)^ method using normal melanocytes as calibrator.

The article "FGF5 is expressed in melanoma and enhances malignancy in vitro and in vivo" was published in 2017. Journal: Oncotarget.

### Forced overexpression of FGF5

FGF5 cDNA was obtained from Geneservice (BC074858, Cambridge, UK) and subcloned into the bicistronic expression vector pIRES2-GFP (Clontech, Mountain View, CA, USA) with EcoRI. The control plasmid contained only GFP. Cells were transfected with Fugene 6 and selected with G418 for 2-3 weeks. Then GFP-positive cells were collected by flow cytometry and cultivated for subsequent experiments.

### FGF5 silencing

Melanoma cells were transduced with 4 different FGF5-targeting short hairpin (sh)RNA lentiviruses and one scrambled shRNA control virus (Sigma, St Louis, MO, USA) as per the manufacturer´s instructions. Stably transduced cells were selected with puromycin and expanded. For experiments using siRNA, cells were transfected with 10 nM FGF5 siRNA or non-silencing control (Santa Cruz Biotechnology, Dallas, TX, USA) using RNAi Max (Thermo Scientific) as transfection reagent.

### Growth curve

Melanoma cells (1×10^5^ cells per well) were seeded into 6-well plates in medium with 10% FBS. Cell number was determined every 2^nd^ day for 8 days with a Casy cell counter (Roche Innovatis AG, Bielefeld, Germany).

### Clonogenic assay

Melanoma cells (3×10^3^ cells per well) were seeded into 6-well plates in medium with 10% FBS and colony formation was assessed after 14 days as described after staining with crystal violet [25]. For analysis of FGF5-treated cells, recombinant human FGF5 (PeproTech, Rocky Hill, NJ, USA) was added every third day. For analyzing the effect of FGF5-targeting siRNA, cells were transfected with siRNA on day 1 and 7 after seeding.

### Transwell invasion assay

Transwell chambers with 8 μm pore size membranes (BD Biosciences, Franklin Lakes, NJ, USA) were coated with collagen and 4×10^4^ cells per well were seeded into the upper chamber. After 72 h, cells that had migrated to the bottom of the lower chamber were stained with crystal violet and evaluated colorimetrically.

### Reporter gene assay

Melanoma cells (3×10^5^ cells per well) were seeded into 6-well plates and on the next day transfected with the plasmids pFA2-ELK1 and pFA-luc (Path Detect ELK1 trans reporting system, Agilent, Santa Clara, CA, USA) for assaying MAPK activity, NFAT-luc (Clontech) for assaying NFAT activity and phACT-359luc [42] for assaying STAT3 activity. For normalization, all wells were co-transfected with a plasmid expressing mCherry. After 24 h (VM1, VM21) or 48 h (VM8), mCherry fluorescence was recorded on a Typhoon Trio imager (GE Healthcare, Little Chalfont, UK) and luciferase activity was determined with the One Glow luciferase assay (Promega, Fitchburg, WI, USA) and a Tecan Infinite M200 Pro microplate reader (Tecan, Männedorf Switzerland).

The article "FGF5 is expressed in melanoma and enhances malignancy in vitro and in vivo" was published in 2017. Journal: Oncotarget.

### Tumor formation *in vivo*

Cells were grown in 75 cm^2^ dishes and 1×10^6^ cells in 50 μl 20% matrigel/PBS were subcutaneously injected into the rear flanks of severe combined immunodeficient (SCID) BALB/c recipient mice (females, 4 per group, Harlan Winkelmann, Borchen, Germany). Tumor formation was measured periodically by palpation and tumor size was determined using a vernier caliper. Tumor volume was calculated as: (smaller diameter^2^ x larger diameter) / 2. Mice were sacrificed after 40 days and tumors were excised and processed for histology. All experiments were carried out according to the Austrian and FELASA guidelines for animal care and protection and were approved by the institutional ethics board (BMWF-66.009/0140-ii/3b/2011).

### Immunohistochemistry

Xenografts were excised and processed for histology as described [12]. A human melanoma tissue array was purchased from US Biomax (Rockville, MD, USA). Slides were deparaffinized and heat-mediated antigen retrieval was done in 0.01 M citrate buffer. The goat polyclonal FGF5 antiserum (AF-237-NA; R&D Systems, Minneapolis, MN, USA) and the Ki67 mouse monoclonal antibody (clone MIB-1, Dako Glostrub, Denmark) were used at dilutions of 1:200 and 1:100, respectively. Bound antibodies on tissue sections were detected with the UltraVision LP detection system (Thermo Scientific). Color development was done with 3,30-diaminobenzidine and counterstaining with haematoxylin. For negative controls, the primary antibodies were replaced by non-immune serum. The percentage of Ki67-positive cell nuclei was assessed in four mice per group in three high-power fields per mouse.

### Apoptosis detection

Slides were deparaffinized and incubated with trypsin (10x, Sigma, 37°C) for 1 h. After 8 min permeabilization with Triton X100 (0.1% in PBS), cells were washed and incubated with TUNEL (terminal deoxynucleotidyl transferase dUTP nick end labeling) mix from the in situ cell death detection kit (Roche, Mannheim, Germany, 50 μl/well) for 1 h at 37°C in the dark and mounted in Vectashield mounting medium containing DAPI (Vector Laboratories, Peterborough, UK). Images were taken on an Olympus BX60 fluorescence microscope with a Nikon DS Fi1 camera. The ratio between DAPI-positive and TUNEL-positive nuclei from 3 images per mouse and >350 cells per image was counted to calculate the percentage of apoptotic cells.

The article "FGF5 is expressed in melanoma and enhances malignancy in vitro and in vivo" was published in 2017. Journal: Oncotarget.

### Immunoblotting of secreted FGF5

Cells (3×10^5^) were seeded in 6-wells and on the next day medium was changed to serum-free medium. After 48 h supernatant was collected and total protein precipitated with 4 volumes of aceton. Pellets were dissolved in protein lysis buffer and proteins subjected to immunoblotting as described [25] with a rabbit polyclonal FGF5 antibody (FL-268, Santa Cruz Biotechnology, 1:200) and a rabbit monoclonal beta 2 microglobulin (b2mg) antibody (Cell Signaling Technology, 1:1000).

### Analysis of angiogenesis

For detection of tumor-infiltrating murine blood vessels, slides were processed as described for Ki67 immunostaining above and incubated with rabbit anti-mouse CD31 antibody (Thermo Scientific, dilution 1:100). Detection of bound antibody was done with the UltraVision LP detection system and AEC (3-amino-9-ethylcarbazole) substrate. Intratumoral microvessel density was counted as described [43].

### Statistical analysis

For all *in vitro* analyses, data are presented as mean and SEM of at least three experiments. Statistical significance between two groups and more than two groups was analyzed with Student's t-test and one-way ANOVA, respectively. P < 0.05 was considered statistically significant.

### Abbreviations

FFPE: formalin-fixed paraffin-embedded
FGF: fibroblast growth factor
FGFR: fibroblast growth factor receptor
GFP: green fluorescent protein
HCC: hepatocellular carcinoma
IHC: immunohistochemistry
MAPK: Mitogen-activated protein kinase
NFAT: nuclear factor of activated T-cells
NSCLC: non-small cell lung cancer
PI3K: phosphatidylinositol-3 kinase
PLC: phospholipase C
RTK: receptor tyrosine kinase
sh: short hairpin
STAT: signal transducer and activator of transcription
TCGA: the Cancer Genome Atlas
TUNEL: terminal deoxynucleotidyl transferase dUTP nick end labeling

## References

[1] Johnson DB, Sosman JA (2015). Therapeutic Advances and Treatment Options in Metastatic Melanoma. JAMA Oncol.

[2] Lee CS, Thomas CM, Ng KE (2017). An Overview of the Changing Landscape of Treatment for Advanced Melanoma. Pharmacotherapy.

[3] Dummer R, Goldinger SM, Paulitschke V, Levesque MP (2015). Curing advanced melanoma by 2025. Curr Opin Oncol.

[4] Acevedo VD, Ittmann M, Spencer DM (2009). Paths of FGFR-driven tumorigenesis. Cell Cycle.

[5] Powers CJ, McLeskey SW, Wellstein A (2000). Fibroblast growth factors, their receptors and signaling. Endocr Relat Cancer.

[6] Weiss J, Sos ML, Seidel D, Peifer M, Zander T, Heuckmann JM, Ullrich RT, Menon R, Maier S, Soltermann A, Moch H, Wagener P, Fischer F (2010). Frequent and focal FGFR1 amplification associates with therapeutically tractable FGFR1 dependency in squamous cell lung cancer. Sci Transl Med.

The article "FGF5 is expressed in melanoma and enhances malignancy in vitro and in vivo" was published in 2017. Journal: Oncotarget.

[7] Elbauomy Elsheikh S, Green AR, Lambros MB, Turner NC, Grainge MJ, Powe D, Ellis IO, Reis-Filho JS (2007). FGFR1 amplification in breast carcinomas: a chromogenic in situ hybridisation analysis. Breast Cancer Res.

[8] Cappellen D, De Oliveira C, Ricol D, de Medina S, Bourdin J, Sastre-Garau X, Chopin D, Thiery JP, Radvanyi F (1999). Frequent activating mutations of FGFR3 in human bladder and cervix carcinomas. Nat Genet.

[9] Gauglhofer C, Sagmeister S, Schrottmaier W, Fischer C, Rodgarkia-Dara C, Mohr T, Stattner S, Bichler C, Kandioler D, Wrba F, Schulte-Hermann R, Holzmann K, Grusch M (2011). Up-regulation of the fibroblast growth factor 8 subfamily in human hepatocellular carcinoma for cell survival and neoangiogenesis. Hepatology.

[10] Miura S, Mitsuhashi N, Shimizu H, Kimura F, Yoshidome H, Otsuka M, Kato A, Shida T, Okamura D, Miyazaki M (2012). Fibroblast growth factor 19 expression correlates with tumor progression and poorer prognosis of hepatocellular carcinoma. BMC Cancer.

[11] Rodeck U, Becker D, Herlyn M (1991). Basic fibroblast growth factor in human melanoma. Cancer Cells.

[12] Schelch K, Hoda MA, Klikovits T, Munzker J, Ghanim B, Wagner C, Garay T, Laszlo V, Setinek U, Dome B, Filipits M, Pirker C, Heffeter P (2014). Fibroblast growth factor receptor inhibition is active against mesothelioma and synergizes with radio- and chemotherapy. Am J Respir Crit Care Med.

[13] Zhan X, Bates B, Hu XG, Goldfarb M (1988). The human FGF-5 oncogene encodes a novel protein related to fibroblast growth factors. Mol Cell Biol.

[14] Hebert JM, Rosenquist T, Gotz J, Martin GR (1994). FGF5 as a regulator of the hair growth cycle: evidence from targeted and spontaneous mutations. Cell.

[15] Suzuki S, Kato T, Takimoto H, Masui S, Oshima H, Ozawa K, Suzuki S, Imamura T (1998). Localization of rat FGF-5 protein in skin macrophage-like cells and FGF-5S protein in hair follicle: possible involvement of two Fgf-5 gene products in hair growth cycle regulation. J Invest Dermatol.

[16] Taniguchi F, Harada T, Sakamoto Y, Yamauchi N, Yoshida S, Iwabe T, Terakawa N (2003). Activation of mitogen-activated protein kinase pathway by keratinocyte growth factor or fibroblast growth factor-10 promotes cell proliferation in human endometrial carcinoma cells. J Clin Endocrinol Metab.

[17] Sundberg JP, Rourk MH, Boggess D, Hogan ME, Sundberg BA, Bertolino AP (1997). Angora mouse mutation: altered hair cycle, follicular dystrophy, phenotypic maintenance of skin grafts, and changes in keratin expression. Vet Pathol.

The article "FGF5 is expressed in melanoma and enhances malignancy in vitro and in vivo" was published in 2017. Journal: Oncotarget.

[18] Higgins CA, Petukhova L, Harel S, Ho YY, Drill E, Shapiro L, Wajid M, Christiano AM (2014). FGF5 is a crucial regulator of hair length in humans. Proc Natl Acad Sci U S A.

[19] Kornmann M, Ishiwata T, Beger HG, Korc M (1997). Fibroblast growth factor-5 stimulates mitogenic signaling and is overexpressed in human pancreatic cancer: evidence for autocrine and paracrine actions. Oncogene.

[20] Hanada K, Perry-Lalley DM, Ohnmacht GA, Bettinotti MP, Yang JC (2001). Identification of fibroblast growth factor-5 as an overexpressed antigen in multiple human adenocarcinomas. Cancer Res.

[21] Lu T, Sathe SS, Swiatkowski SM, Hampole CV, Stark GR (2004). Secretion of cytokines and growth factors as a general cause of constitutive NFkappaB activation in cancer. Oncogene.

[22] Fang F, Chang RM, Yu L, Lei X, Xiao S, Yang H, Yang LY (2015). MicroRNA-188-5p suppresses tumor cell proliferation and metastasis by directly targeting FGF5 in hepatocellular carcinoma. J Hepatol.

[23] Allerstorfer S, Sonvilla G, Fischer H, Spiegl-Kreinecker S, Gauglhofer C, Setinek U, Czech T, Marosi C, Buchroithner J, Pichler J, Silye R, Mohr T, Holzmann K (2008). FGF5 as an oncogenic factor in human glioblastoma multiforme: autocrine and paracrine activities. Oncogene.

[24] Albino AP, Davis BM, Nanus DM (1991). Induction of growth factor RNA expression in human malignant melanoma: markers of transformation. Cancer Res.

[25] Metzner T, Bedeir A, Held G, Peter-Vorosmarty B, Ghassemi S, Heinzle C, Spiegl-Kreinecker S, Marian B, Holzmann K, Grasl-Kraupp B, Pirker C, Micksche M, Berger W (2011). Fibroblast Growth Factor Receptors as Therapeutic Targets in Human Melanoma: Synergism with BRAF Inhibition. J Invest Dermatol.

[26] Uribe P, Wistuba II, Gonzalez S (2003). BRAF mutation: a frequent event in benign, atypical, and malignant melanocytic lesions of the skin. Am J Dermatopathol.

[27] Ibrahim N, Haluska FG (2009). Molecular pathogenesis of cutaneous melanocytic neoplasms. Annu Rev Pathol.

[28] Wang Y, Becker D (1997). Antisense targeting of basic fibroblast growth factor and fibroblast growth factor receptor-1 in human melanomas blocks intratumoral angiogenesis and tumor growth. Nat Med.

[29] Halaban R, Kwon BS, Ghosh S, Delli Bovi P, Baird A (1988). bFGF as an autocrine growth factor for human melanomas. Oncogene Res.

[30] Han X, Xiao Z, Quarles LD (2015). Membrane and integrative nuclear fibroblastic growth factor receptor (FGFR) regulation of FGF-23. J Biol Chem.

[31] Perotti V, Baldassari P, Bersani I, Molla A, Vegetti C, Tassi E, Dal Col J, Dolcetti R, Anichini A, Mortarini R (2012). NFATc2 is a potential therapeutic target in human melanoma. J Invest Dermatol.

The article "FGF5 is expressed in melanoma and enhances malignancy in vitro and in vivo" was published in 2017. Journal: Oncotarget.

[32] Nesbit M, Nesbit HK, Bennett J, Andl T, Hsu MY, Dejesus E, McBrian M, Gupta AR, Eck SL, Herlyn M (1999). Basic fibroblast growth factor induces a transformed phenotype in normal human melanocytes. Oncogene.

[33] Blackwell C, Sherk C, Fricko M, Ganji G, Barnette M, Hoang B, Tunstead J, Skedzielewski T, Alsaid H, Jucker BM, Minthorn E, Kumar R, DeYoung MP (2015). Inhibition of FGF/FGFR autocrine signaling in mesothelioma with the FGF ligand trap, FP-1039/GSK3052230. Oncotarget.

[34] Marek LA, Hinz TK, von Massenhausen A, Olszewski KA, Kleczko EK, Boehm D, Weiser-Evans MC, Nemenoff RA, Hoffmann H, Warth A, Gozgit JM, Perner S, Heasley LE (2014). Nonamplified FGFR1 is a growth driver in malignant pleural mesothelioma. Mol Cancer Res.

[35] Rizvi S, Yamada D, Hirsova P, Bronk SF, Werneburg NW, Krishnan A, Salim W, Zhang L, Trushina E, Truty MJ, Gores GJ (2016). A Hippo and Fibroblast Growth Factor Receptor Autocrine Pathway in Cholangiocarcinoma. J Biol Chem.

[36] Mitchell SM, Ross JP, Drew HR, Ho T, Brown GS, Saunders NF, Duesing KR, Buckley MJ, Dunne R, Beetson I, Rand KN, McEvoy A, Thomas ML (2014). A panel of genes methylated with high frequency in colorectal cancer. BMC Cancer.

[37] Sonvilla G, Allerstorfer S, Stattner S, Karner J, Klimpfinger M, Fischer H, Grasl-Kraupp B, Holzmann K, Berger W, Wrba F, Marian B, Grusch M (2008). FGF18 in colorectal tumour cells: autocrine and paracrine effects. Carcinogenesis.

[38] Seo HR, Jeong HE, Joo HJ, Choi SC, Park CY, Kim JH, Choi JH, Cui LH, Hong SJ, Chung S, Lim DS (2016). Intrinsic FGF2 and FGF5 promotes angiogenesis of human aortic endothelial cells in 3D microfluidic angiogenesis system. Sci Rep.

[39] Rathjen J, Lake JA, Bettess MD, Washington JM, Chapman G, Rathjen PD (1999). Formation of a primitive ectoderm like cell population, EPL cells, from ES cells in response to biologically derived factors. J Cell Sci.

[40] Pirker C, Holzmann K, Spiegl-Kreinecker S, Elbling L, Thallinger C, Pehamberger H, Micksche M, Berger W (2003). Chromosomal imbalances in primary and metastatic melanomas: over-representation of essential telomerase genes. Melanoma Res.

[41] Mathieu V, Pirker C, Schmidt WM, Spiegl-Kreinecker S, Lotsch D, Heffeter P, Hegedus B, Grusch M, Kiss R, Berger W (2012). Aggressiveness of human melanoma xenograft models is promoted by aneuploidy-driven gene expression deregulation. Oncotarget.

[42] Cvijic H, Bauer K, Loffler D, Pfeifer G, Blumert C, Kretzschmar AK, Henze C, Brocke-Heidrich K, Horn F (2009). Co-activator SRC-1 is dispensable for transcriptional control by STAT3. Biochem J.

[43] Dome B, Paku S, Somlai B, Timar J (2002). Vascularization of cutaneous melanoma involves vessel co-option and has clinical significance. J Pathol.

The article "FGF5 is expressed in melanoma and enhances malignancy in vitro and in vivo" was published in 2017. Journal: Oncotarget.

[44] Colaprico A, Silva TC, Olsen C, Garofano L, Cava C, Garolini D, Sabedot TS, Malta TM, Pagnotta SM, Castiglioni I, Ceccarelli M, Bontempi G, Noushmehr H (2016). TCGAbiolinks: an R/Bioconductor package for integrative analysis of TCGA data. Nucleic Acids Res.

